# Computer-Aided Diagnosis of COVID-19 CT Scans Based on Spatiotemporal Information Fusion

**DOI:** 10.1155/2021/6649591

**Published:** 2021-03-03

**Authors:** Tianyi Li, Wei Wei, Lidan Cheng, Shengjie Zhao, Chuanjun Xu, Xia Zhang, Yi Zeng, Jihua Gu

**Affiliations:** ^1^College of Optoelectronic Science and Engineering, Soochow University, Suzhou, Jiangsu 215006, China; ^2^MeBotX Intelligent Technology (Suzhou) Co. Ltd., Suzhou, Jiangsu 215000, China; ^3^The Department of Radiology, The Second Hospital of Nanjing, Affiliated Hospital Nanjing University of Chinese Medicine, Nanjing, Jiangsu 210003, China; ^4^The Department of Tuberculosis, The Second Hospital of Nanjing, Affiliated Hospital Nanjing University of Chinese Medicine, Nanjing, Jiangsu 210003, China; ^5^The Center for Global Health, School of Public Health, Nanjing Medical University, Nanjing, Jiangsu 211166, China

## Abstract

Coronavirus disease (COVID-19) is highly contagious and pathogenic. Currently, the diagnosis of COVID-19 is based on nucleic acid testing, but it has false negatives and hysteresis. The use of lung CT scans can help screen and effectively monitor diagnosed cases. The application of computer-aided diagnosis technology can reduce the burden on doctors, which is conducive to rapid and large-scale diagnostic screening. In this paper, we proposed an automatic detection method for COVID-19 based on spatiotemporal information fusion. Using the segmentation network in the deep learning method to segment the lung area and the lesion area, the spatiotemporal information features of multiple CT scans are extracted to perform auxiliary diagnosis analysis. The performance of this method was verified on the collected dataset. We achieved the classification of COVID-19 CT scans and non-COVID-19 CT scans and analyzed the development of the patients' condition through the CT scans. The average accuracy rate is 96.7%, sensitivity is 95.2%, and F1 score is 95.9%. Each scan takes about 30 seconds for detection.

## 1. Introduction

From the end of 2019, coronavirus disease (COVID-19) has disseminated around the world and become a global challenge, leading the World Health Organization to declare the COVID-19 outbreak a pandemic [1–3]. Up to now, no clinically approved therapeutic is available for treatment [4]. The findings showed that COVID-19 virus spreads from person to person. It is necessary to block the spread of COVID-19 by isolating patients, tracing, and isolating close contacts [5]. Therefore, a study of a timely and effective diagnosis method that can quickly screen as many scans as possible is needed.

At present, the diagnosis of COVID-19 mainly depends on the nucleic acid kit for reverse transcription-polymerase chain reaction (RT-PCR) to determine the presence of viral nucleic acid [6]. As a disease diagnosis, especially infectious diseases, the final diagnosis still needs to rely on the etiology. Although RT-PCR is considered the gold standard for COVID-19 diagnosis, there are still some influencing factors, such as the degree of standardization of sample collection and the time of sample collection [7]. Also, whether RT-PCR can detect COVID-19 depends on the viral load. If the sampling site does not contain viruses nor has a low viral load, the nucleic acid test will be prone to false negatives.

Since some cases have imaging features, but nucleic acid detection has hysteresis, medical imaging methods (such as chest X-ray (CXR) and computer tomography (CT)) can play a significant role in the diagnosis of COVID-19 [8, 9]. Besides, nucleic acid testing can only diagnose whether a patient has COVID-19. But it cannot judge the condition, while medical imaging can [10]. For patients with COVID-19, accurate monitoring of disease progression is a vital component of disease management. For suspected cases, such as close contacts of COVID-19 patients whose nucleic acid test is negative, imaging can be used for monitoring [8, 9].

In general, medical imaging methods are effective means to diagnose COVID-19 and monitor disease progression. Real-time analysis of the patient's condition is necessary for doctors to determine effective treatment methods. Accurate and quantitative analysis of the disease can help doctors prescribe the right medicine.

Traditional imaging diagnosis depends on the experience of doctors. COVID-19 is a new type of infectious disease, and current research has summarized the imaging characteristics of this type of disease [9]. Usually, one CT scan contains multiple slices. It takes 5–15 minutes for doctors to examine one CT scan. Repetitive work will cause the doctor's mental fatigue. Rapid and large-scale detection and screening cannot be performed. Doctors can only use subjective judgments to analyze the development of patients' conditions, which cannot be intuitive and quantitative.

In recent years, deep learning has achieved great success in the area of computer vision, which provides new solutions to the automated processing of medical images [11–15]. Artificial intelligence technologies, especially deep learning tools, can be developed to help radiologists perform data classification, quantification, and trend analysis. If the CT scan shows the possibility of disease, the case can be marked for further examination by a radiologist or clinician for possible treatment or quarantine. Computer-aided diagnosis (CAD) system based on CT scans can help doctors diagnose COVID-19 and better understand disease development. It is worth noting that CAD technology cannot replace doctors or other medical professionals, the final diagnosis must be judged by professionals.

In summary, nucleic acid detection has a certain misdiagnosis rate and hysteresis and requires a certain detection time [10]. CT scans of the lungs can provide rapid auxiliary diagnosis and monitor the condition of the disease. But doctors need to spend a lot of energy to interpret the CT slices, especially in areas with severe epidemics, requiring large-scale rapid screening. In response to the abovementioned problems of the COVID-19 diagnosis and detection, we proposed a method for the assisted diagnosis of COVID-19 based on CT scans. This method is based on the spatiotemporal sequence information of CT scans to realize the detection and analysis of COVID-19 scans. Its contributions are as follows:

1. Using the fast and effective segmentation network LinkNet and training the false positive network for removing lesions based on the DenseNet network structure to achieve accurate segmentation of the lesion area;
2. Combining the characteristics of the spatiotemporal of CT scans, effectively monitoring the disease development, assisting doctors intuitively understanding the condition, and determining the diagnosis and treatment.

Experimental results show that the auxiliary diagnosis method has good detection and classification effects. It can visually display the disease development and assist doctors in clinical diagnosis and treatment.

### 1.1. Related Work

The computer-aided diagnosis system uses imaging, medical image processing technology, and other means combined with computer analysis and calculation to assist in diagnosis. Many applications have been proposed in medical imaging, including segmentation and characterization tasks.

Convolutional neural network (CNN) is developed for the detection of breast cancer [11], brain tumor [12], pulmonary nodules [13], intracranial aneurysm [14], and other diseases [15]. Usually, a two-step approach is adopted, first determining the area of interest and then reducing false positives [15].

Chung et al. [16] gave a more detailed description of the COVID-19 CT scans. These CT scans show an extent of irregular ground-glass opacities that progress rapidly after COVID-19 symptom onset [16, 17]. In the early stage of the disease, CT images show image features of multiple small patches and interstitial changes. Then, it develops multiple ground glass shadows and infiltration shadows of the lungs. In severe cases, lung consolidation may occur, and pleural effusions are rare [18].

Fang et al. [19] compared the sensitivity of chest CT detection with nucleic acid detection by RT-PCR. 51 patients received initial and repeated RT-PCR tests. Their standard is the diagnosis of COVID-19 infection finally confirmed by serial RT-PCR testing. In this patient sample, the detection rate for initial CT (50 of 51 patients (98%); 95% CI: 90%, 100%) was greater than that for first RT-PCR (36 of 51 patients (71%); 95% CI: 56%, 83%). Xie et al. [20] also have reported a lack of sensitivity in the initial RT-PCR test.

Bernheim and Huang [21] studied 121 cases of chest CT studies obtained in the early, middle, and late infections of four centers in China. Studies have shown that the appearance of frosted glass on both sides and surrounding lungs is characteristic of the disease.

Based on these image features shown in Figure 1, a few studies have already reported deep learning to diagnose COVID-19 pneumonia on chest radiograph or CT.

Kassania et al. [22] compared popular deep learning-based feature extraction frameworks for automatic COVID-19 classification. They tested the combination of different deep learning networks combined with machine learning methods for classification. Experimental results show that the DenseNet121 feature extractor with the bagging tree classifier achieved the best performance with 99% classification accuracy.

Fei et al. [23] developed a deep learning- (DL-) based segmentation system with a human-in-the-loop (HITL) strategy to assist radiologists for infection region segmentation. By comparing the automatically divided infection area and the manually divided area, the average similarity coefficient is about 91.6%.

Hemdan et al. [24] developed COVIDX-Net for diagnosing COVID-19 in X-ray Images. The authors conducted a comparative study of different deep learning architectures. The dataset includes 50 X-ray images, divided into 25 non-COVID-19 images and 25 COVID-19 images. Experimental results demonstrated VGG19 and DenseNet201 models achieved the best performance scores among similar models, with F1 scores of 0.89 and 0.91 for non-COVID-19 and COVID-19, respectively. However, the dataset used in the experiment is small.

Gozes et al. [25] presented a system that utilizes 2D and 3D deep learning models. By modifying and adapting existing AI models (RAD Logics Inc., Boston), this study demonstrated that rapidly developed AI-based image analysis can achieve high accuracy in the detection of coronavirus as well as quantification and tracking of disease burden.

Basu et al. [26] proposed a new concept called domain extension neural network to solve the problem that the available COVID-19 data are rare and not easy to train. The overall accuracy was 95.3% ± 0.02.

Maghdid et al. [27] used the deep learning method and transfer learning strategies to diagnose COVID-19 automatically. The structure is a combination of CNN structure and an improved AlexNet structure. The improved architecture accuracy reaches 94.10% on the X-rays and CT slice dataset.

Hasan et al. [28] presented a promising technique for predicting COVID-19 patients from the CT scan using CNN. The approach based on DenseNet is the updated CNN architecture in the present state to detect COVID-19. The results outperformed 92% accuracy, with 95% recall.

At present, there are some studies of lung CT detection, most of them use a single CT slice, such as [28], and the sequence features of CT scans are not fully utilized. In fact, during the doctor's diagnosis process, the doctor will not judge based on a single slice. Especially when the slice is in doubt, the slices before and after will affect the judgment. What's more, in addition to the study of different patients, the analysis of CT scans of one patient during the treatment also plays an important role for the doctor to judge the development of the disease and the effectiveness of the treatment method.

## 2. Methods

This study was mainly divided into two parts: COVID-19 classification and detection experiment based on sequence feature of CT scan to classify and detect; COVID-19 volume measurement experiment based on the CT scans obtained during one patient's treatment. By measuring the volume of the lesion and fusing time information of the CT scans, we can intuitively quantify the development of the disease and analyze the patient's condition. The overall flow chart is shown in Figure 2.

### 2.1. Preprocessing

#### 2.1.1. Dataset

This experiment collected 445 lung CT scans of COVID-19 and 63 healthy lung CT scans from Nanjing Infectious Diseases Hospital (the Second Hospital of Nanjing). The COVID-19 CT scans were from 142 patients. Each patient took several times of chest CT scans during their treatment, and the CT slice thickness was 0.625 mm to 1.250 mm. Nanjing Infectious Diseases Hospital is a designated hospital for COVID-19 in Jiangsu Province. The use of data was approved by the Ethics Society and was only used for this experimental study. The patient's information was kept confidential. The 445 cases we collected included various stages of disease development, and each scan contains hundreds of slices. Also, we selected 170 lung CT scans randomly from the online public dataset LUNA16 [29] for the COVID-19 classification experiment as negative samples to form the dataset. So, the total datasets contain 445 COVID-19 scans and 233 non-COVID-19 scans. The data from LUNA16 were reprocessed, the HU value was adjusted to the range of −1200∼600, it was set to −1200 if it is less than −1200, it was set to 600 if it is greater than 600, and then it was normalized to 0 ∼255. The CT slice size is 512 ^∗^ 512 pixels.

#### 2.1.2. Experiment Condition

The Windows-based computer system used for this work had an Intel(R) Core(TM) i7-8700K 3.7 GHz processor with 16 GB RAM. The training and testing process of the proposed architecture for this experiment was implemented in Python using Pytorch backend as the deep learning framework backend running on NVIDIA GeForce GTX 1080 Ti GPU.

#### 2.1.3. Evaluation Criteria

Taking into account the unevenness of the data, a single verification indicator may not be able to summarize the performance of the algorithm. We utilized a variety of common evaluation metrics such as precision (PRE), recall (REC), accuracy (AUC), and F1 score (F1).

  Precision: among all the samples judged to be correct, it is the correct proportion
  Recall: among all the positive samples, it is the proportion of correct judgment
  F1 score: comprehensive performance indicators are concerned about the accuracy of positive samples and their recall
  TP (true positive): the number of instances that correctly predicted
  TN (true negative): the number of instances that incorrectly predicted
  FP (false positive): the number of negative instances that predicted correctly
  FN (false negative): the number of negative instances that predicted correctly all evaluation metrics calculated as follows:

(1) $$\begin{array}{c} \text{precision}=\frac{\text{TP}}{\text{TP}+\text{FP}}, \end{array}$$

(2) $$\begin{array}{c} \text{recall}=\frac{\text{TP}}{\text{TP}+\text{FN}}, \end{array}$$

(3) $$\begin{array}{c} \text{accuracy}=\frac{\text{TP}+\text{TN}}{\text{TP}+\text{TN}+\text{FP}+\text{FN}}, \end{array}$$

(4) $$\begin{array}{c} \text{F}1\text{ score}=2*\frac{\text{recall}*\text{precision}}{\text{recall}+\text{precision}}. \end{array}$$

### 2.2. COVID-19 Classification

The rapid COVID-19 detection was based on the sequence features of COVID-19 CT scans. The flow chart is shown in Figure 3. There are three steps in the experiment: lung area segmentation, lesion area segmentation, and classification. The lesion area segmentation step includes the false positive screening of the lesion area. The lung area and the lesion area obtained during the detection process can be used in lesion volume measurement experiments.

#### 2.2.1. Lung Segmentation

In the original CT slice, there are other surrounding tissue parts besides the lung area we need. Too much redundant information is in the picture, which will interfere with training and testing. Therefore, we first segmented the lung area.

Previous studies have shown that U-net can be trained end-to-end from very few images and achieve excellent performance [30]. So, the U-net has become the most popular base network widely used in biomedical image segmentation. To speed up the training and processing of the network, we chose the LinkNet network structure. The LinkNet network is a variant of the U-net [31] and is a typical encoder-decoder structure. The encoder is used for feature extraction and dimension reduction of the input images, while the decoder will restore the feature information into an image. The encoder and decoder connection structure is shown in Figure 4. The encoder structure uses residual connections. The feature map after introducing the residual is more sensitive to the changes in output, and the gradients are easier to train. The learning features of encoder block *i* from shallow to deep can be expressed as follows:

(5) $$\begin{array}{c} EB_{i}=E_{i2}\left(E_{i1}\left(e_{i}\right)+e_{i}\right)+E_{i1}\left(e_{i}\right)+e_{i},\;i=1,2,3,4, \end{array}$$

where *E*_*i*1_(*e*_*i*_) is the result after weighted convolution, *EB*_*i*_ is the output of the encoder block *i*, and also the input of the encoder block *i*+1, *e*_*i*_ is the input of the encoder block *i*.

The encoder block *i* and decoder block *i* are directly connected to improve accuracy and reduce processing time [31].

(6) $$\begin{array}{c} DB_{i}=D_{i}\left(d_{i}\right), \end{array}$$

(7) $$\begin{array}{c} d_{i-1}=DB_{I}+e_{i}. \end{array}$$

The decoder block structure shown in Figure 4 can be expressed as equation (6), where the *D*_*i*_(*d*_*i*_) is the result after weighted convolution, *DB*_*i*_ is the output of the decoder block *i*, and *d*_*i*_ is the input of the decoder block *i*. The input of encoder block *i* − 1 can be expressed as formula (7).

The training steps of the lung segmentation model are shown in Figure 5. Using pretrained models for testing, we found that when the CT slice contains ground glass shadow in the lung area, especially the ground glass shadow in the lung edge area, the model could not segment the lung area accurately. To optimize the network, take the CT slices from 20 scans of COVID-19 and 10 scans of non-COVID-19 randomly as the input, supplement, and correct the label of lung region obtained by the test to get their integral lung label images. Then, the 20 scans in pretrained and 30 scans in the test with their label images are used as the input of the segmentation network to improve the robustness and reliability of the model. Finally, we obtained a retrained lung segmentation model and the lung area of other slices obtained through the model test.

In order to verify the effectiveness of the segmentation method used in this article, 10 scans were randomly selected for lung segmentation test, of which 6 were COVID-19 scans and 4 were non-COVID-19 scans. Among them, the COVID-19 CT scans contain imaging features, and the lesions are distributed on the periphery of both lungs. These 10 scans were only tested for segmentation, and the model was not modified by them, so they continued being used in the next experiment. The results are shown in Table 1, where M1 is the initial training model, and M2 is the model trained by adding modified supplementary marks and unprocessed images. IOU (intersection over union) value is used for evaluation, as shown in equation (8), where Area_mask_ is the area of the marked target area, Area_test_ is the area of the tested target area. By supplementing the training data, we improved the lung area division and divided the ground glass shadow in the edge area correctly.

(8) $$\begin{array}{c} \text{IOU}=\frac{{\text{Area}}_{\text{mask}}\cap {\text{ Area}}_{\text{test}}}{{\text{Area}}_{\text{mask}}\cup {\text{Area}}_{\text{test}}}. \end{array}$$

#### 2.2.2. Lesion Segmentation

The lung segmentation network training scans were also used as the input of the lesion segmentation network. The lesions of the COVID-19 are mainly ground glass shadows. We invited many professional doctors from the Second Hospital of Nanjing to mark the lesion. Based on the abovementioned test for segmentation network, the lesion segmentation network also applies the LinkNet model.

The lung segment was tested using the trained lesion segmentation network, and the lesion regions in the rest of 628 scans were segmented, and then we cropped each lesion area. The test process of lesion segmentation is shown in Figure 6. We found some negative image pieces in the segmented lesion area, which needs to be screened for false positives.

Since DenseNet performed excellently in object recognition [32], it has also been proved useful for COVID-19 image classification in previous research [22, 24], so we use this network to train false positives screening. There may be multiple lesion areas detected in one slice, so it was necessary to cut into lesion area blocks according to the mask area and determine whether each lesion area block was a real lesion.

Due to the limited data, we selected 10 positive scans and 11 negative scans randomly for training. Then, we resized the lesion area blocks to 64 ^∗^ 64. Even during the detection of positive sections, some negative lesions may be included. So, we needed to filter them out before training. To improve the generalization of the training model, we used data augmentation for small samples. The data augmentation technique is a widely used method for training models to increase training benefits and decrease the effect of network regularization. All the data were augmented by horizontal and vertical flip, width and height shift, and rotation with angles of 90°,180°, and 270°, so that the number of training data expanded about fivefold.

#### 2.2.3. Feature Extraction and Classification

The decision tree method in machine learning was used for final classification. In the previous steps, we obtained the lesion area in each CT slice. But it is not reliable to detect one slice to represent the entire scan. Therefore, we chose 8 overall features of the CT scan, the features are shown in Table 2. Then, we used the decision tree for training classification and testing.

The training and testing datasets have 607 scans, except the 50 scans used in lung segmentation and the other 21 scans used in lesion segmentation, including 415 COVID-19 scans and 192 non-COVID-19 scans. The training set and test set were divided according to a ratio of 6 : 4.

#### 2.2.4. Model Parameters

The parameters used in each model for training are shown in Table 3.

### 2.3. COVID-19 Volume Measurement

In CT scan diagnosis, doctors can analyze the patients' condition according to the lesion changes. COVID-19 has different imaging manifestations due to the disease development, and the most intuitive manifestation is the change in lesion volume. By analyzing all the CT scans of one patient, we could judge the disease development according to the changes in the lesion volume.

In this COVID-19 volume measurement experiment, according to the CT scans during the patient's treatment, based on time information of each scan, the lesion volume was calculated to assist doctors in quantifying the condition and analyzing the development. In the classification experiment, we have already obtained the lung area and the lesion area of the patient image for this experiment.

As the lung volume changes with breathing, it is impossible to simply obtain an accurate volume of the lung, and the corresponding lesion volume cannot be accurately measured. To simplify the calculation, do not perform three-dimensional reconstruction of the image sequence, using the image sequence directly to convert the calculation of the three-dimensional lesion volume into the calculation of the two-dimensional lesion area. Calculating the sum of the pixel area of the lung area and the lesion area of all slices in each CT scan to obtain the proportion of the lesion volume and the lung volume, as shown in formula (9), where Area_Lesion_ is the sum of the pixel area of the lesion area, Area_Lung_ is the sum of the pixel area of the lung area. By calculating the ratio, we can solve the problem that the basic difference of lung volume between different patients makes it impossible to use the same quantitative standard to judge.

(9) $$\begin{array}{c} \text{Per}=\frac{\text{Area}\_\text{Lesion}}{\text{Area}\_\text{Lung}}. \end{array}$$

## 3. Results and Discussion

### 3.1. Classification Result

We tested on the collected dataset using the abovementioned experimental methods. Due to data imbalance, we referenced the five-fold cross-validation method and divided the remaining 607 data into 5 groups, and each group of data is composed as shown in Table 4. P_Num is the number of COVID-19 CT scans, N_Num is the number of non-COVID-19 CT scans, and A_Num is the number of total CT scans.

Randomly taking three groups of data for training and the remaining two groups of data for testing, the accuracy, precision, sensitivity, and F1-score are calculated. A total of 10 datasets were formed for training and testing. The results of the 10 sets of data are shown in Table 5. We use 95% CI (confidence interval) on the obtained datasets, we get the average accuracy of 94.4% (95%CI: 91.6%–97.2%), precision 96.7% (95%CI: 94.5%–98.9%), recall 95.2% (95%CI: 92.5%–97.9%), and *F*1-score 96.0%.

Partial entry in Table 5 is in the format (*µ* ± *σ*) where *µ* is the average value, and 95%CI is (*µ*−*σ*) to (*µ*+*σ*).

At the same time, we tested the time used for each part of the algorithm. Due to the different number of sequence images, the time used for detection will change accordingly. In the test, when the average number of slices in the test scan is 103, the average time of the key part of the algorithm is shown in Table 6.

According to the abovementioned experimental steps, the automatic diagnosis system of COVID-19 based on CT scan was integrated, and we made a software of COVID-19 auxiliary diagnosis based on C++ and Libtorch. The time of the software to detect one CT scan is calculated. In 60 CT scans, the average number of images is 100, and the average detection time per scan is 28.78 s.

### 3.2. Volume Measurement Result

The scans of 142 patients from the hospital were collected in this experiment, and each patient contains images with varying times of detections.

Take one patient's scans as an example. As shown in Figure 7, it shows that the patient has 12 times of detection between January and April. The abscissa in Figure 7 shows the detection date of the CT scans. The ordinate shows the proportion of the lung area and the lesion area in the scan. For the convenience of the display, it was plotted as a percentage. Doctors could visually see the changes in the lesion volume according to the data line chart shown in Figure 7. The patient has gone through a period of rapid development from the onset of COVID-19 and hospitalization and has gradually improved after treatment. In general, doctors can intuitively judge the disease development and treatment effect based on the measurement and analysis of the patients' CT scans.

## 4. Conclusions

In conclusion, the rapid and effective diagnosis and disease development analysis of COVID-19 is important in the current situation where COVID-19 is still spreading. Nucleic acid detection has false negative and hysteresis. Also, it cannot judge the severity of the condition. Lung CT scans can provide auxiliary diagnosis and monitor the disease progression. To assist doctors in realizing rapid diagnosis and rapid interpretation of lung CT scans, this paper proposed an automatic COVID-19 detection method based on spatiotemporal information fusion. It analyzes the spatial characteristics of CT scans to assist doctors in COVID-19 diagnosis and fuses time information of the scans to assist doctors in quantifying the patient's condition. We achieved the classification of COVID-19 and non-COVID-19 on the collected datasets. We use the LinkNet network to train the lung and lesion segmentation network and the DenseNet network to train the false positive screening network. Considering that the relationship of the features between the CT slices will affect the judgment of classification, we extracted the sequence features of CT scans instead of the features of one single slice. The decision tree method is used for classification and by quantifying the lesion volume of the CT scan and fusing time information, we realized the computer-aided diagnosis of COVID-19.

Experimental results show the following:

1. The result on the obtained dataset gets an average accuracy of 94.4%, precision of 96.7%, recall of 95.2%, and F1 score of 96.0%.
2. Analysis of the CT scans from the patient during his treatment can intuitively quantify the disease development and analyze the disease development trend.
3. The lung segmentation and lesion segmentation training methods in this study could be used for segmentation recognition of other diseases (such as tumors). The lung segmentation network could also be used for preliminary data processing of diagnosis of other lung diseases. The method could also be extended to other kinds of medical images.

However, it has to be acknowledged that our classifier may not be capable of distinguishing non-COVID interstitial pneumonia from COVID interstitial pneumonia, whose CT lesion phenotypes are similar. How to distinguish between COVID-19 and other pneumonia makes our follow-up research directions.

## Figures and Tables

**Figure 1:** The lesion area of COVID-19 on the CT images.

**Figure 2:** Overall experiment flow chart.

**Figure 3:** Flowchart of the proposed framework for computer-aided COVID-19 diagnosis. (a) Image preprocessing. (b) Training lung segmentation, training lesion segmentation, and training DenseNet for false positive screening. (c) Extract features for classification.

**Figure 4:** The structure of LinkNet.

**Figure 5:** Training process of the lung segmentation model.

**Figure 6:** Test process of lesion segmentation.

**Figure 7:** The trend of the lesion volume of one patient's multiple detection.

**Table 1:** Test results of lung segmentation model.

Cases	Label	M1-IOU	M2-IOU
Eg1	P	0.967	0.978
Eg2	P	0.934	0.942
Eg3	P	0.906	0.921
Eg4	P	0.973	0.979
Eg5	P	0.926	0.926
Eg6	P	0.924	0.952
Eg7	N	0.978	0.979
Eg8	N	0.983	0.984
Eg9	N	0.825	0.825
Eg10	N	0.882	0.884

**Table 2:** Features of decision tree.

Feature	Definition
Slice_Num	The number of slices with the lesion area
Lesion_AreaSum	The total area of lesion area
Lesion_AeraMax	The largest lesion area
Lesion_MaxPosition	The position of the slice with the largest lesion in the CT scan
Slice_NumPercent	The ratio of the number of slices with lesions to the total number of slices
Lesion_MaxPercent	The ratio of the largest lesion area to the lung area of that slice
Lesion_SumPercent	The ratio of the sum of lesion area to the sum of lung area in the slice with lesion
Lesion_AllSumPercent	The ratio of the total area of the lesion to the total area of the lung

**Table 3:** Parameters of models.

Model	Parameter	Value
Segmentation model	Batch size	16
	Epoch	100
	Loss function	BCEWithLogitsLoss
	Optimizer	Adam
	Learning rate	10^−3^

False positive screening model	Batch size	128
	Epoch	200
	Learning rate	5 ^∗^ 10^−3^
	Loss function	Cross-entropy loss
	Optimizer	SGD

Decision tree model	Criterion	“Gini”
	Class_weight	“Balanced”
	Splitter	“Best”

**Table 4:** Composition of 5 groups of data.

Set	A-Num	P-Num	N-Num
X1	122	83	39
X2	122	83	39
X3	122	83	39
X4	121	83	38
X5	120	83	37
ALL	607	415	192

**Table 5:** The test result of the 10 datasets.

Data	Test	AUC (95%CI)	Pre (95%CI)	Rec (95%CI)	F1
Dataset1	X4X5	93.8 ± 3.0	95.2 ± 2.7	95.9 ± 2.5	0.955
Dataset2	X3X5	95.0 ± 2.7	98.1 ± 1.7	94.6 ± 2.8	0.963
Dataset3	X3X4	95.5 ± 2.6	96.4 ± 2.3	97.0 ± 2.1	0.967
Dataset4	X2X5	93.0 ± 3.2	96.9 ± 2.2	92.8 ± 3.3	0.948
Dataset5	X2X4	94.7 ± 2.8	95.8 ± 2.5	96.4 ± 2.3	0.961
Dataset6	X2X3	92.6 ± 3.3	96.8 ± 5.5	92.2 ± 3.3	0.944
Dataset7	X1X5	95.0 ± 2.7	96.4 ± 2.3	96.4 ± 2.3	0.964
Dataset8	X1X3	96.3 ± 2.7	97.6 ± 2.3	97.0 ± 2.3	0.973
Dataset9	X1X2	94.7 ± 2.4	97.5 ± 1.9	94.6 ± 2.1	0.960
Dataset10	X1X4	95.1 ± 2.8	96.4 ± 2.0	96.4 ± 2.8	0.964
Avg.		94.6 ± 2.8	96.7 ± 2.2	95.3 ± 2.7	0.960

**Table 6:** Algorithm time for each part.

Algorithm part	Time (s)
Lung segmentation	5.259
Lesion segmentation	4.727
Remove false positives	4.189
Feature extraction	6.961
Decision tree classification	0.082
Total	21.218

## Data Availability

The COVID-19 CT image data used to support the findings of this study have not been made available because they involve patient privacy.
